The article "The Role for HNF-1β-Targeted Collectrin in Maintenance of Primary Cilia and Cell Polarity in Collecting Duct Cells" was retracted in 2023. Reasons: manipulated images; errors in the images; errors in the text; duplicated images.

# The Role for HNF-1β-Targeted Collectrin in Maintenance of Primary Cilia and Cell Polarity in Collecting Duct Cells

**DOI:** 10.1371/journal.pone.0000414

**Published:** 2007-05-02

**Authors:** Yanling Zhang, Jun Wada, Akihiro Yasuhara, Izumi Iseda, Jun Eguchi, Kenji Fukui, Qin Yang, Kazuya Yamagata, Thomas Hiesberger, Peter Igarashi, Hong Zhang, Haiyan Wang, Shigeru Akagi, Yashpal S. Kanwar, Hirofumi Makino

**Affiliations:** 1 Department of Medicine and Clinical Science, Okayama University Graduate School of Medicine, Okayama, Japan; 2 Department of Nephrology, Third Hospital Hebei Medical University, Shijiazhuang, China; 3 Department of Metabolic Medicine, Graduate School of Medicine, Osaka University, Osaka, Japan; 4 Division of Endocrinology, Diabetes, and Metabolism, Beth Israel Deaconess Medical Center, Harvard Medical School, Boston, Massachusetts, United States of America; 5 Department of Internal Medicine and Division of Basic Science, University of Texas Southwestern Medical Center, Dallas, Texas, United States of America; 6 Renal Division, Institute of Nephrology, Peking University First Hospital, Peking University, Beijing, China; 7 Northwestern University, The Feinberg School of Medicine, Department of Pathology, Chicago, Illinois, United States of America; University of Hong Kong, China

## Abstract

Collectrin, a homologue of angiotensin converting enzyme 2 (ACE2), is a type I transmembrane protein, and we originally reported its localization to the cytoplasm and apical membrane of collecting duct cells. Recently, two independent studies of targeted disruption of collectrin in mice resulted in severe and general defects in renal amino acid uptake. Collectrin has been reported to be under the transcriptional regulation by HNF-1α, which is exclusively expressed in proximal tubules and localized at the luminal side of brush border membranes. The deficiency of collectrin was associated with reduction of multiple amino acid transporters on luminal membranes. In the current study, we describe that collectrin is a target of HNF-1β and heavily expressed in the primary cilium of renal collecting duct cells. Collectrin is also localized in the vesicles near the peri-basal body region and binds to γ-actin-myosin II-A, SNARE, and polycystin-2-polaris complexes, and all of these are involved in intracellular and ciliary movement of vesicles and membrane proteins. Treatment of mIMCD3 cells with collectrin siRNA resulted in defective cilium formation, increased cell proliferation and apoptosis, and disappearance of polycystin-2 in the primary cilium. Suppression of collectrin mRNA in metanephric culture resulted in the formation of multiple longitudinal cysts in ureteric bud branches. Taken together, the cystic change and formation of defective cilium with the interference in the collectrin functions would suggest that it is necessary for recycling of the primary cilia-specific membrane proteins, the maintenance of the primary cilia and cell polarity of collecting duct cells. The transcriptional hierarchy between HNF-1β and PKD (polycystic kidney disease) genes expressed in the primary cilia of collecting duct cells has been suggested, and collectrin is one of such HNF-1β regulated genes.

## Introduction

In a previous study, we identified a member of angiotensin converting enzyme (ACE) gene family, collectrin, by its up-regulation in a mouse model of partial nephrectomy [1], which is a long-standing model for the progressive renal diseases. Collectrin is a type I transmembrane protein and we originally reported its localization to the cytoplasm and apical membrane of collecting duct cells. It is a homologue of ACE2 and identified in immediate proximity of the *ace2* locus. ACE2 may be a chimeric protein emerging from the duplication of two genes, having homology with ACE at the catalytic domain and homology with collectrin in the membrane proximal domain[2]. Unlike ACE and ACE2, collectrin lacks N-terminal active dipeptidyl carboxypeptidase catalytic domain, and thus its biology has not been well-established. Recently, two independent studies of targeted disruption of *collectrin* in mice resulted in a severe and general defects in renal amino acid uptake[3], [4]. Collectrin is demonstrated at the luminal side of brush border membranes of proximal tubules and the deficiency of collectrin is associated with reduction of multiple amino acid transporters, such as B0AT1, rBAT, B^0,+^AT[4], XT3s1/ST1, XT2, XT3 and EAAC1[3], on luminal membranes.

We and others have described the expression of collectrin in pancreatic β cells and collectrin is identified as a target of hepatocyte nuclear factor-α (HNF-1α)[5], [6]. Targeted disruption of HNF-1α resulted in diabetes and a renal phenotype with Fanconi syndrome characterized by glucosuria, phosphaturia, calciuria and aminoaciduria[7]. Localization of HNF-1α in proximal tubules and similar renal phenotype in collectrin and HNF-1α knockout mice suggested that the expression of collectrin in proximal tubules is transcriptionally regulated by HNF-1α. In contrast to HNF-1α, the renal-specific inactivation of HNF-1β develops polycystic kidney disease, and renal cyst formation is accompanied with a drastic defect in the transcriptional activation of several polycystic kidney disease (PKD)-related genes, such as *Umod, Pkhd1, Pkd2 and Tg737/Polaris* [8]. Similarly, mutations in HNF-1β gene are seen in the autosomal dominant disorder MODY5 (maturity-onset diabetes mellitus of the young, type 5)[9] and MODY5 patients present type 2 diabetes and develop congenital kidney abnormalities including simple cysts, polycystic kidneys, cystic dysplasia and glomerulocystic kidney disease. The expression of collectrin and HNF-1β in collecting duct cells suggested that collectrin is also regulated by HNF-1β and play roles in renal cyst formation or sodium and water handling. Collectrin knockout mice are lacking in the phenotype of diabetes, hypertension and renal cystic formation[3], [4]; however, it can be speculated that collectrin play a role in the pathophysiology of pancreatic β cells and collecting duct cells because many other genes, such as ACE2, may compensate the action of collectrin in the gene disruption studies. For instance, overexpression of collectrin in INS1-E cells and insulin promoter driven collectrin transgenic mice enhanced glucose-induced insulin exocytosis. Collectrin binds to SNARE (soluble N-ethylmaleiamide-sensitive factor attachment protein receptor) complex by interacting with snapin, a SNAP-25 (synaptosomal-associated protein of 25 kDa) binding protein, and facilitates the SNARE complex formation[10]. Thus, collectrin facilitates the insulin excytosis by regulating the SNARE complex formation. Based on line of evidences, we hypothesized that collectrin plays a role in vesicle trafficking of various apical membrane proteins in a polarized manner by which we can easily explain why the recruitment of multiple amino acid transporters at apical membranes is disturbed by collectrin deficiency.

Here, we investigated the role of collectrin using collecting duct cell lines (mIMCD-3 cells), Ksp-cadherin promoter driven dominant-negative HNF1β mutant (DN-HNF1β) [11] and HNF-1β deletion mutant lacking C-terminal domain (HNF1βΔC) transgenic mice[12]. We have demonstrated that HNF-1β controls the transcriptional activities of collectrin. Furthermore, collectrin is preferentially associated with primary cilium and is shown to play a role in primary cilium formation, cell polarity and maturation revealed by siRNA experiments. We also demonstrated that the expression of collectrin on vesicles in peri-basal body region and its ability to bind to SNARE complex by interacting with snapin and to form complex with ciliary proteins, such as polycistin-2 and polaris. Collectrin may mediate specific vesicle transport, upon docking deliver the integral membrane proteins to ciliary plasmalemma, and maintain the primary cilia and cell polarity in collecting duct cells.

## Materials and Methods

### Animals

Ksp-cadherin promoter regulated dominant-negative HNF1β mutant (DN-HNF1β) transgenic mice[11] and HNF-1β deletion mutant lacking C-terminal domain (HNF1βΔC) transgenic mice[12] were produced by the University of Texas Southwestern Transgenic Core Facility.

### Preparation of stable mIMCD3 cell lines overexpressing collectrin

The nucleotide sequence encoding *myc* epitope, GAACAAAAACTCATCTCAGAAGAGGATCTG, was introduced into human collectrin cDNA in frame distal to the signal sequence by PCR and then subcloned into pcDNA3.1 to generate expression vector pcDNA3.1-*myc*-collectrin. mIMCD3 cells (ATCC) were transfected with pcDNA3.1-*myc*-collectrin plasmid using Lipofectamine 2000 reagent (Invitrogen). Stable transformants were selected by the treatment of Geneticin (300 µg/ml, Sigma).

### Cloning of 5′ flanking promoter region of rat, mouse, and human collectrin and transcriptional elements scanning

The 5′ flanking promoter regions of rat, mouse, and human collectrin genes were cloned into pT7 blue vector (Invitrogen) using Genome Walker Kit (Clontech) as described previously[13]. Following which the DNA sequences for transcriptional elements were identified by using TRANSFAC database of weighted matrices of transcription factor binding sites.

### Generation of collectrin antibodies

Polyclonal antibodies were raised in rabbits against the mixture of synthetic peptides derived from mouse collectrin amino acid sequence, AFSMRKVPNREATEISH (55-71) and AAEVQSAIRKNRNRINS (98-114) using custom polyclonal antibody production service (Asahi Techno Glass Corp., Tokyo, Japan). The specific binding to both peptides and the titers were confirmed by ELISA (enzyme-linked immunosorbent assay) (Asahi Techno Glass Corp).

### Electrophoretic mobility shift assay (EMSA)

Plasmids encoding the full length of human HNF-1α and HNF1β were prepared by PCR from human kidney cDNA and cloned into pcDNA3.1(+) vector (Invitrogen). Nuclear proteins were extracted using Nuclear Extract Kit (Active Motif) from mIMCD3 cells with or without pcDNA3.1/HNF-1α transfection. EMSAs were performed with Dig Gel Shift Kit 2nd generation (Roche). Nuclear protein (2 µg) was incubated with digoxygenin-labelled oligonucleotide containing HNF-1 binding site of the human collectrin gene (5′-GATGGGTGTTAATCATTAAACCTTT-3′). The DNA-protein complexes were loaded on 5% polyacrylamide non0denaturing gels. The monoclonal HNF-1α and HNF-1β antibody (Transduction Laboratories) was used for supershift assays.

### Transient transfection and luciferase-reporter assay

Promotor region segments of human collectrin containing putative HNF-1 binding site were generated by PCR and cloned into pGL3 basic reporter vector (Promega)[13]. mIMCD3 cells were co-transfected with 0.5–1.0 µg of pcDNA3.1/HNF-1α and/or pcDNA3.1/HNF-1β vectors, 0.5 µg of pGL3-collectrin reporter and 10 ng of pBIND vector using Lipofectamine 2000 reagent. 48 hours following transfection, the cells were lysed in 500 µl passive lysis buffer (Promega), firefly and renilla luciferase activities were measured using the Dual-Luciferase Reporter Assay System (Promega). The luciferase activity was expressed as the ratio of firefly and renilla luciferase activity.

### Western blotting

Subcellular fractions of SD rat and CD-1 mouse kidneys were prepared by differential centrifugation as described[14]. Briefly, an initial spin was carried out at 800 *g* to remove nuclei and incompletely homogenized cellular debris. The supernatant was spun at 17,000 *g* for 20 min to pellet the plasma membranes (PM); the 17,000 *g* supernatant was subjected to a high-speed centrifugation (200,000 *g*) for 60 min in a Beckman 70Ti rotor to sediment the intracellular vesicle membranes (VM). The protein lysates of mIMCD3 cells, whole kidney and its subcellular fraction were subjected to SDS-PAGE and transferred to Nylon membranes. The membranes were treated with specific antibodies (1∶1000 dilution), such as mouse anti-HNF-1α and HNF-1β (Transduction Laboratories), polyclonal anti-SNARE associated protein (snapin) (Synaptic Systems, Göttingen, Germany), rabbit anti-rat aquaporin-2, goat anti-polycystin-2, rabbit anti-epidermal growth factor receptor (EGFR)(Santa Cruz Biotechnology, Santa Cruz, CA), and rabbit anti-collectrin, overnight at 4°C and followed by the treatment with secondary antibodies conjugated with horseradish peroxidase (1∶20000 dilution)[15].

### Enzymatic deglycosylation

The mouse medullary total protein was extracted and used for N-deglycosylation analysis. N-Glycosidase F Deglycosylation Kit was used following vendor's instructions (Roche). About 500 µg protein was incubated with 10 U of O-Glycosidase (Roche) for 3 h at 37°C. The reaction mixtures were then subjected to Western blot analyses.

### Yeast two-hybrid screening and tandem affinity tag (TAP) purification

Collectrin cDNA encoding intracellular domain was subcloned to pGBKT7 bait vector and mouse kidney library was constructed using pGADT7-Rec vector. Yeast two-hybrid screening was performed according to the manufacturer's protocol (BD Biosciences Clontech). The collectrin cDNA containing full coding region without N-terminal signal sequence was cloned into pNTAP (Stratagene) and transiently transfected into mIMCD3 cells. Final purified proteins were analyzed with SDS-PAGE and Coomassie blue staining. The major bands were isolated and subjected to MALDI-TOF MS (mass spectrometry).

### Immunoprecipitation studies of mIMCD-3 cell lines

mIMCD3 cells were lysed in RIPA buffer (20 mM Tris-HCl, pH 7.4, 100 mM NaCl, 1 mM CaCl_2_, 1 mM MgCl_2_, and 1% Triton X-100) with protease inhibitor cocktail (Roche Diagnostics Co., Basel, Switzerland). The lysates were centrifuged at 12,000 *g* for 30 minutes at 4°C and the supernatants were incubated with the preimmune sera and protein A-Sepharose CL-4B (Amersham Biosciences, GE Healthcare, Uppsala, Sweden). Immunoprecipitations were performed by adding 10 µl of specific sera and 80 µl of protein-A Sepharose CL-4B to 0.5 ml of supernatants further incubated overnight at 4°C on a rocking platform. The immunoprecipitated complexes were dissolved in a gel-loading buffer (50 mM Tris-HCl, pH 6.8, 2% SDS, 10% glycerol, 100 mM DTT, and 0.1% bromophenol blue), subjected to SDS-PAGE under the reducing condition, and electroblotted onto Hybond P PVDF membranes (Amersham Biosciences, Piscataway, NJ). They were immunoblotted with specific antibodies (1∶100 to 1∶1000) overnight at 4°C and followed with the secondary antibodies conjugated with horseradish peroxidase (1∶20000). Finally, the filters were immersed in ECL Plus Western Blotting Detection Reagents (Amersham), and then exposed to Hyperfilm ECL (Amersham). Rabbit anti-rat snapin (Synaptic Systems), goat anti-human SNAP-23 (synaptosomal-associated protein 23 kDa), goat anti-human syntaxin-4, goat anti-polycystin-2 (Santa Cruz), rabbit anti-polaris, rabbit γ-actin (Novus Biologicals, Littleton, CO), rabbit anti-tropomyosin (CHEMICON, Temecula, CA) antibodies were used for immunoprecipitation and Western blot analyses. Normal rabbit and goat IgGs were used for negative controls of immunoprecipitation.

### Experiments with collectrin specific siRNA

siTrio targeting mouse collectrin (NM_020626;5′-CCATAAGAATGAACAGAATT-3′, 5′-GCAGAAGACAAGTGTGAAATT-3′, 5′-CAACAATAGACCACTGAAATT-3′)(Collectrin siRNA) and siTrio negative control cocktail containing double stranded RNAs (5′-ATCCGCGCGATAGTACGTATT-3′, 5′-TTACGCGTAGCGTAATACGTT-3′ and 5′-TATTCGCGCGTATAGCGGTTT-3′)(CON siRNA) were purchased from DHARMACON and transfection of mIMCD3 cells was carried out with Lipofectamine 2000 reagent. Following experiments were performed 24 hours after the transfection. Cells in chamber slides were stained with mouse anti-PCNA monoclonal antibody (BD Transduction Lab) using R.T.U Vectastain Universal Quick kit (Vector Laboratories, Burlingame, CA, U.S.A.), apoptosis was evaluated with the DeadEndTM Colorimetric TUNEL System (Promega), and cell viability was assessed by MTT based colorimetric assay for the cell proliferation and viability (Roche). Western blot analyses and immunofluorescence were carried out using rabbit anti-EGFR (epidermal growth factor receptor) polyclonal antibody (1∶2000 dilution, Santa Cruz). For immunofluorescnce, cells grown in chamber slides were fixed in 4% paraformaldehyde for 30 minutes at 4°C, and then permeabilized with 0.1% Triton X-100 in PBS for 3 min if necessary. After blocking in 8% BSA in PBS for 1 hour at room temperature, cells were incubated at 4°C overnight with the primary antibodies diluted in 1% BSA. After washing for 5 minutes with PBS, cells were incubated for 1 hour with fluorescein isothiocyanate (FITC) or tetramethyl rhodamine isothiocyanate (TRITC)-conjugated secondary antibodies. Rabbit anti-collectrin, mouse γ-tubulin, mouse anti-acetylated α-tubulin, mouse anti-Golgi 58K (Sigma), mouse anti-disulfide isomerase (Stressgen, Bictoria, Canada), rabbit anti-EGFR (Santa Cruz) were used. The cells were then examined by a confocal laser scanning microscope, Laser Scanning System LSM 510 (Carl Zeiss, Jena, Germany). Immunoelectron microscopy was performed using rabbit anti-collectrin antibody (1∶300 dilution) and goat anti-rabbit IgG conjugated with 15 µm colloidal gold (Amersham) as secondary antibody (1∶20 dilution)[16].

### Quantification of primary cilium numbers and length in mIMCD3 cells

Immunofluorescence images of primary cilia double stained with collectrin and acetylated tubulin were generated using LSM510 confocal microscope system (Zeiss). Percentage of the cells with visually detectable cilia was evaluated in ∼200 mIMCD3 cells and measurements of cilia length were determined using Zeiss LSM image browser software.

### Organ culture and antisense experiments

Embryonic kidneys were harvested from pregnant Crl:CD-1 (ICR) mice at day 13 of gestation (E13)[17]. Antisense-phosphorothioated oligodeoxynucleotides (ODNs) of collectrin, HNF1α, HNF1β and a nonsense ODN were prepared as follows; 5′-CTCTGAAGAGGTATTCTTGATCCGT-3′, 5′-TCAGGTCCCCTCGACTCCACCGCA-3′ and 5′-ATAGTCGTCGCCGTCCTCTGAGCCCTC-3′, and 5′-TAATGATATAATGATTGTAATGATAGTAGT-3′. E13 metanephroi were maintained in an organ culture containing 12.5 µg/ml of epidermal growth factor (EGF). The antisense and nonsense ODNs were added to the culture medium daily at concentrations ranging from 1.5 to 2.5 µM for 4 days, and the metanephroi were subjected to quantitative real-time PCR. PCR was optimized and carried out on an ABI PRISM 7000 sequence detection system (Applied Biosystems) using ABsolute^TM^ QPCR SYBR Green Mix (ABgene, Rochester, NY). For each gene, the denaturation at 95°C for 15min was followed by 40 cycles of denaturation at 95°C for 15 sec, annealing at 60°C for 30 sec and extension at 72°C for 30 sec. Gene specific primers for *collectrin* (Genbank accession #AF178085), *Pkhd1* (NM_153179), *Pkd2* (NM_008861), *Umod* (NM_009470), *Tg737/Polaris* (NM_009376) and β-actin (NM_007393) were as follows: *collectrin* forward (5′-GCAATTGCACTACTGGTTCTAT CTG-3′), *collectrin* reverse (5′-TCCACTCCAGGTGGTCCTTT-3′), *Pkhd1* forward (5′-TG ACCTTTTCTAGAT TGGCTGTCTT-3′), *Pkhd1* reverse (5′-GT CCTTGATCGAGCTGTAA AATTAG-3′), Pkd2 forward (5′-TGAGCGTGAGCATCAACAGAT-3′), *Pkd2* reverse (5′-T GGTAAAGAGCTGT GTTCCAAGTC-3′), *Umod* forward (5′-AGGTGTCCAGGCCTCAGTG T-3′), *Umod* reverse (5′-GGAAACAACAGCAGCCAGATG-3′), *Tg737/Polaris* forward (5′-TGCCT GGGACAGATGAA CCT-3′), *Tg737/Polaris* reverse (5′-AGGGCCCAGTGGATCCA-3′), β-actin forward (5′-GGCGCT TTTGACTCAGGATT-3′), β-actin reverse (5′-GGGATGTTTGCTCC AACCAA-3′).

### Data analysis

Data were expressed as mean±s.e.m. Multiple groups were compared by analysis of variance (ANOVA). Two-group analysis was performed by t-test.

## Results

### Collectrin is transcriptionally regulated by HNF-1β in collecting duct cells

To investigate the transcriptional regulation of collectrin gene, ∼500-bp of the 5′ flanking promoter region of rat collectrin gene was cloned. Transcriptional elements and consensus sequence of HNF-1 binding site were identified[13]. Comparison of the rat, human and mouse collectrin genes using GenBank data revealed that HNF-1 binding site was conserved. RT-PCR and Western blot analyses revealed that HNF-1β was expressed in mIMCD3 cells, while HNF-1α was not detected. HNF-1α mRNA and protein were detected in mIMCD-3 cells transfected with pcDNA3.1/HNF-1α (**Figure 1a**). The binding of HNF-1 to the putative promoter elements in mIMCD3 cells was confirmed by electrophoretic mobility shift assay (EMSA) (**Figure 1a**). The incubation of DNA probes of putative HNF-1 binding site with nuclear extracts from non-transfected or pcDNA3.1/HNF-1α transfected mIMCD3 cells revealed specific DNA-protein complex formation. The collectrin gene promoter was inserted into promoterless pGL3-Basic vector, where the transcription of the luciferase gene was driven by the collectrin promoter. This construct was cotransfected into mIMCD3 cells with pcDNA3.1/HNF-1α and/or pcDNA3.1/HNF-1β vectors. As shown in **Figure 1b**, cotransfection with pcDNA3.1/HNF-1α and/or pcDNA3.1/HNF-1β vectors accentuated luciferase activity in a dose dependent manner. These results indicated that HNF-1α and HNF-1β regulate the transcription of collectrin gene via HNF-1 binding consensus sequence present in its promoter.

**Figure 1:** Transcriptional regulation of collectrin gene by HNF-1β. *Panel a:* Western blot analysis, RT-PCR and electrophoretic mobility shift assay (EMSA). Endogenous mRNA expression of HNF-1β but not HNF-1α in mIMCD3 cells is detected by Western blot analysis and RT-PCR. The specific binding of HNF-1β and HNF-1α to putative binding site is indicated by antibody mediated supershift (arrow). *Panel b:* Luciferase reporter gene assay. The mIMCD3 cells are co-transfected with pcDNA3.1/HNF-1α and/or pcDNA3.1/HNF-1β with pGL3-collectrin reporter and pBIND vector. A dose dependent increase in the reporter activity is observed (n = 6, *p<0.05 and **p<0.01 versus pcDNA3.1(+) treated control) *Panel c:* Western blot analyses of collectrin using whole kidney lysates of DN-HNF1β transgenic mouse. In two transgenic mouse founders, the expression of DN-HNF1β mutant transgene tagged with V5 and FLAG epitope is indicated by percentage of highest expression, 6% and 100%. (Western blot analysis using anti-FLAG antibody, n = 3 separate measurements, *p<0.05 and **p<0.01 versus non-transgenic littermate indicated by 0%) *Panel d:* Localization of collectrin and HNF-1β deletion mutant protein in epithelia lining the cyst shown by immunofluorescence microscopy. Collectrin is visualized as red, HNF-1β deletion mutant with V5 tag as green, and nuclei as blue. Arrows indicate the absence of collectrin expression on the apical surface of epithelial cells where HNF-1β deletion mutant product is expressed in the nucleus. Scale bar, 20 µm.

### Dominant negative mutations of HNF-1β inhibited collectrin expression in vivo

HNF-1β is expressed in renal collecting duct cells both in tissues and cell lines. Whole kidney membrane fractions from dominant-negative HNF-1β mutant (DN-HNF1β) transgenic mice[11] were extracted to confirm transcriptional regulation of collectrin by HNF-1β. DN-HNF1β transgenic founders with lower expression of transgene had smaller decrease in collectrin, and the transgenic founder with higher transgene expression exhibited remarkable decrease in collectrin revealed by Western blot analysis using whole kidney lysates **(** **Figure 1c** **)**. Next, we examined the expression of collectrin in collecting ducts in HNF-1β deletion mutant lacking C-terminal domain tagged with V5 epitope (HNF1βΔC) transgenic mice[12]. The kidney tissue sections from transgenic founders, chimeric mice with wild type HNF-1β and HNF-1β deletion mutant, were stained with collectrin antibody (red) and V5 antibody (green) (**Figure 1d**) and nuclei were counterstained blue with 4′-6-diamidino-2-phenylindole. The luminal expression of collectrin was absent on the epithelial cells (arrows) in which HNF1βΔC was highly expressed in the nuclei (green); while collectrin was apparently expressed in surrounding normal collecting duct cells that did not express HNF1βΔC transgene product (blue).

### Collectrin localizes to primary cilia

Plasma and vesicle membrane fractions from mouse and rat renal medulla were associated with aquapirin-2 and snapin, respectively (**Figure 2a**). The molecular weight of collectrin, ∼40 kDa, was similar in mouse, rat and human, both in plasma and vesicle membrane fractions. Collectrin is a glycosylated protein since the predicted molecular weight from amino acid sequence was ∼26 kDa. Deglycosylation with N- and O-glycosidase resulted in the reduction in molecular weight, *i.e.* 30 kDa and 35 kDa, respectively (**Fig. 2b**). Next, subcellular localization of collectrin by immunofluorescence was investigated. Focal planes of single mIMCD3 cell were obtained; the nuclear focal plane indicated that collectrin localized in cytoplasm, and the apical focal plane revealed the presence of collectrin on apical plasma membrane (**Figure 2c**).

**Figure 2:** Subcellular localization of collectrin in kidney tissues and mIMCD3 cells. *Panel a:* Western blot analyses of snapin, aquaporin-2 and collectrin, isolated from plasma membrane (PM) and vesicle membrane (VM) fractions. Collectrin antibody detected a single band of ∼40 kDa. *Panel b:* N-glycosidase (N) and O-glycosidase (O) treatment generates ∼30 kDa and ∼35 kDa respective bands. *Panel c:* Immunoreactivity of collectrin is detected by confocal microscopy; five layers (1 to 5) are shown and collectrin is seen in cytoplasm (2 to 5 cuts) and apical membrane (1 cut). *Panel d:* Apical view of mIMCD3 cells. Collectrin (green) and acetylated α-tubulin (red), a primary ciliary marker, are depicted. *Panel e:* Higher magnification shows that acetylated α-tubulin (red) and collectrin (green) co-localize. *Panel f:* Collectrin (green) is seen surrounding the γ-tubulin, a marker for the basal body (red). *Panel g:* Immunoelectron microscopy shows gold particles localized mainly in microvesicles around the basal body of the primary cilium (arrow heads), whereas few gold particles are observed at the peripheral region of proximal centriole. Scale bars, 20 µm for panels c, d, e, and f and 500 nm for panel g.

Scanning the mIMCD3 cells using confocal microscopy from basal cell attachment to apical top and re-construction of three-dimensional images indicated that primary cilia displayed intense immunoreactivities. Double staining of anti-acetylated α-tubulin, marker for primary cilia, and anti-collectrin antibodies confirmed that collectrin expression was concentrated in primary cilia (**Figure 2d**). Higher magnification of the apical focal plane clearly showed the co-localization of collectrin and acetylated α-tubulin on primary cilium (**Figure 2e**). Collectrin immunoreactivities (green) were seen surrounding the ciliary basal body, the latter is visualized with anti-γ-tubulin antibody (red)(**Figure 2f**). Similarly, immunoelectron microscopy revealed that gold particles were associated with the vesicles adjacent to the basal bodies, while they were not integrated into the basal body microtubule structures. Gold particles were also located at ciliary membranes surrounding the microtubules, whereas few gold particles were observed at the peripheral region of the centriole (**Figure 2g**).

### Cilia formation is disrupted by collectrin siRNA treatment

To demonstrate the role of collectrin in cilia formation, stable mIMCD3 cell lines over-expressing collectrin (collectrin stable) were generated. All 4 cell lines revealed ∼3-fold over-expression compared with control pcDNA3.1 stably transfected mIMCD3 cells (mIMCD3 cells) (**Figure 3a**). The siRNA treatment significantly suppressed collectrin expression in mIMCD3 cells, while the control siRNA had no effect (**Figure 3b**). Confocol microscopy also revealed that collectrin was over-expressed in collectrin stable cells and knocked down by siRNA revealed by confocol microscopy (**Figure 3c**). The fully polarized mIMCD3 cells were associated with single primary cilia, and the cilia formation was not disturbed in control siRNA treated cells or collectrin stable cell lines (**Figure 3d**). However, primary cilia were absent in ∼40% of the cells treated with collectrin siRNA (**Figures 3d and 3e**). In addition, morphometric analyses of the existing primary cilia indicated that mIMCD3 cells transfected with siRNA had shorter or stunted primary cilia compared with those of control siRNA treated cells (**Figures 3d and 3f**). By electron microscopy (**Figure 3g**), the treatment of siRNA resulted in various abnormalities of primary cilia, *e.g.* disorganization of 9+0 microtubular structure of basal bodies (arrow head), bulging basal bodies (arrow), and stunted shaft projection (asterisk).

**Figure 3:** Primary cilium formation in mIMCD3 cells. *Panel a:* Expression of collectrin in mIMCD3 cells over-expressing collectrin (n = 4; clone 11, 13, 15 and 18) and mIMCD3 cells stably transfected with pcDNA3.1(+) (n = 2; clone c1 and c2)(mIMCD3 cells). (*p<0.05 versus mIMCD3 cells) *Panel b:* Western blot analysis of collectrin in mIMCD3 cells treated with control siRNA (CON-siRNA) or Collectrin siRNA. (Data represent 3 independent experiments, *p<0.01 versus CON-siRNA) *Panel c:* Immunofluorescence of collectrin in mIMCD3 cells, CON-siRNA and Collecrin siRNA treated cells, and Collectrin stable cells. *Panels d & e:* mIMCD3 cells double-stained with collectrin (green) and acetylated α-tubulin (red). Cilia are present in every polarized cell, but ∼40% of cells are without detectable cilia with the treatment of collectrin siRNA. AV, apical view. (n = 300 from separate three experiments, *p<0.05 versus CON-siRNA) *Panel f:* Cilium length is also reduced in cells after collectrin siRNA transfection (∼4.5 µm) compared with CON-siRNA group (∼7.8 µm). (n = 300 from three independent experiments, *p<0.05 versus CON-siRNA) *Panel g:* Electron micrographs of mIMCD3 cells treated with CON-siRNA and Collectrin siRNA. Cilium with disorganized microtubule structure (arrow heads), bulging cilium (arrows), and stunted cilium (asterisk) are seen in mIMCD3 cells transfected with Collectrin siRNA. Scale bars, 20 µm for panels c and d and 500 nm for panel g.

### Colocalization of polycystin-2 and collectrin and effects of collectrin siRNA

Since polycyctin-2 reveals ciliary localization and the intracellular trafficking of polycystin-2 is regulated both at the level of the endoplasmic reticulum and the trans-Golgi network, subcellular expression of collectrin and polycystin-2 in mIMCD3 cells was assessed. Inhibition of collectrin expression by siRNA showed negative impact on polycystin-2 protein expression in mIMCD3 cells (**Figure 4a**). Double staining showed that collectrin was fully co-localized with Golgi marker and also partially localized in endoplasmic reticulum (ER) (**Figure 4b**). As expected, collectrin and polycystin-2 colocalized in the cytoplasm of mIMCD3 cells (**Figure 4c**). Apical view by confocal microscopy indicated that polycystin-2 was highly expressed on primary cilia and in the cytoplasm of mIMCD3 cells, whereas polycystin-2 disappeared both in the cilia and cytoplasm of most of the cells transfected with collectrin siRNA (**Figure 4d**).

**Figure 4:** Expression and localization of polycystin-2 in mIMCD3 cells treated with collectrin siRNA. *Panel a:* Western blot analyses show down regulation of polycystin-2 in mIMCD3 cells transfected with collectrin siRNA (Collectrin siRNA). Collectrin expression is not altered in mIMCD3 cells treated with control siRNA (CON-siRNA) and mIMCD3 cells over-expressing collectrin (Collectrin stable). (Data represent 3 independent experiments, *p<0.05 versus CON-siRNA) *Panel b:* mIMCD3 cells double-stained with anti-collectrin antibody and organella markers. Golgi 58K protein (58K-9) (red) and collectrin (green) are co-localized in cytoplasm of mIMCD3 cells. Endoplasmic reticulum (ER) marker, protein disulfide isomerase (red), and collectrin (green) show partial colocalization. *Panel c:* mIMCD3 cells double-stained with polycystin-2 (green) and collectrin (red) showing co-localization. *Panel d:* mIMCD3 cells double-stained with polycystin-2 and acetylated α-tubulin. Polycystin-2 is highly expressed in primary cilia and the apical membrane of mIMCD3 cells, CON-siRNA treated and Collectrin stably transfected cells, whereas polycystin-2 is not detected in the cilia of most of the cells transfected with collectrin siRNA. AV, apical view. Scale bars, 10 µm for panels b, c, and d.

### Collectrin forms complexes with proteins related to vesicle transport and fusion

Further insight into the role of collectrin was investigated by examining protein:protein interactions with ciliary proteins, such as polycyctin-2 and polaris[18]. Co-precipitation of collectrin and polycystin-2 or collectrin and polaris (**Figure 5a**) indicated it forms a complex with polycystin-2 and polaris. Next, collectrin-interacting molecules were identified by yeast two-hybrid system. After screening more than 10^7^ independent clones using intracellular domain of collectrin as bait, snapin, SNAP-25 (synaptosomal-associated protein of 25 kDa) binding protein, was isolated. In a previous study, snapin was also isolated by the yeast two-hybrid system using full-length of collectrin as bait[13]. Snapin is a component of SNARE (soluble N-ethylmaleiamide-sensitive factor attachment protein receptor) and immunoprecipitation study showed collectrin co-precipitated with snapin. In mIMCD3 cells, collectrin also co-precipitated with SNARE proteins, SNAP-23 and syntaxin-4, suggesting collectrin binds to SNARE complex by interacting with snapin (**Fig. 5b**). Further screen of the protein complexes using tandem affinity tag purification and mass spectrometry was performed. Collectrin cDNA lacking N-terminal signal sequence was cloned into pNTAP and transiently transfected into mIMCD3 cells. Purified proteins were analyzed with SDS-PAGE that revealed two major bands. MALDI-TOF MS identified them as nonmuscle myosin heavy chain II-A (myosin heavy polypeptide 9) and γ-actin. Co-immunoprecipitation study revealed collectrin forms the protein complex with γ-actin, myosin II-A, tropomyosin, and polycystin-2 (**Figure 5c**). Although collectrin knockdown alter the intensity and pattern of acetylated α-tubulin, collectrin siRNA treatment did not alter the expression and staining pattern of γ-actin, myosin II-A, and tropomyosin revealed by Western blot analysis and immunofluorescence study (data not shown).

**Figure 5:** Collectrin and interacting proteins. *Panel a:* Immunoprecipitation indicates interaction between collectrin and polycystin-2, and between collectrin and polaris. *Panel b:* Collectrin co-precipitates with snapin, SNAP-23, and syntaxin-4. *Panel c:* Tandem affinity tag purification using collectin as a bait followed by SDS-PAGE and MALDI TOF MS analysis revealed that the major two bands are nonmuscle myosin heavy chain II-A and γ-actin. Immunoprecipitation study shows collectrin, myosin II-A, γ-actin, tropomyosin, and polycystin-2 forms protein complex.

### Collectrin regulates cell proliferation, apoptosis, and polarity

PCNA immunostaining and 5-bromo-2′-deoxyuridine (BrdU) assays showed an increased proliferation activity in mIMCD3 cells transfected with collectrin siRNA, while the stable over-expression of collectrin had no notable effect on cell proliferation (**Figures 6a, 6b and 6c**). To examine the effects of collectrin on apoptosis, TUNEL assay was performed in mIMCD3 cells. The number of apoptotic cells notably increased in mIMCD3 cells transfected by collectrin siRNAs compared with negative control siRNA treated cells. Over-expression of collectrin did not show any alterations in percentage of apoptotic cells (**Figures 6d and 6e**). Although collectrin siRNA-treated mIMCD3 cells underwent apoptosis and revealed proliferation activity, overall viable cell numbers were not altered shown by MTT assay (**Figure 6e**).

**Figure 6:** Proliferation, apoptosis, and mislocalization of epidermal growth factor receptor (EGFR) in mIMCD3 cells treated with collectrin siRNA. *Panels a & b:* Cellular proliferation assessed by proliferating cell nuclear antigen (PCNA) staining. PCNA positive cells increase in mIMCD3 cells treated with collectrin siRNA compared with control siRNA treated cells (CON-siRNA) and mIMCD3 cells over-expressing collectrin (Collectrin stable). *Panel c:* The increased proliferation of cells is observed in collectrin siRNA group by BrdU assay. *Panels d & e:* Apoptosis assay using TdT-mediated dUTP nick end labeling (TUNEL) method. Increased number of apoptotic cells is observed in collectrin siRNA group. *Panel f:* The viability of the cells is not altered in all groups revealed by MTT assay. *Panel g:* Imunofluoresence and confocal micrographs of EGFR. EGFR is observed in basolateral membrane of mIMCD3 cells, control siRNA group, and collectrin stable cells, whereas apical membrane expression of EGFR is detected in collectrin siRNA group. *Panel h:* Western blot analyses of EGFR. EGFR is up-regulated in collectrin siRNA group and down-regulated in cells stably transfected with collectrin. Scale bars, 20 µm for panel f. N = 300 from separate three experiments for panels b, c and e. Data are from 3 independent experiments for panel g, *p<0.05, **p<0.01 versus CON-siRNA.

Since up-regulation and mis-polarization of epidermal growth factor receptor (EGFR) is linked to abnormal cell proliferation, the expression of EGFR was investigated. EGFR was normally expressed on lateral membrane in mIMCD3 cells, and transient transfection with control siRNA or stable trasfection of collectrin gene did not alter the distribution. Besides lateral membrane expression, the EGFR was also seen mis-localized on the apical membrane in the cells treated with collectrin siRNA, a characteristic feature observed in tubular epithelia lining the cysts in human and animal polycystic kidneys[18], [19] (**Figure 6g**). The Western blot analysis revealed that over-expression of collectrin is associated with reduced EGFR, in turn, the repression of collectrin resulted in up-regulated EGFR expression (**Figure 6h**).

### Collectrin antisense ODN treatment of metanephric organ culture

Addition of EGF (12.5 µg/ml) and nonsense ODN resulted in hypertrophy of the fetal kidney without apparent cyst formation (**Figure 7a**-B****) compared with nonsense ODN treated control explants (**Figure 7a-A**). Inclusion of collectrin antisense ODN was associated with formation of cleft-like structure (arrows) in the ureteric bud branches in a dose-dependent manner (**Figures 7a-C and -D**). Addition of HNF-1α antisense ODN into the metanephric organ culture media also resulted in the formation of multiple cleft-like cysts (**Figures 7a-E-F**), while the number or size of the cyst formation were relatively more in the metanephroi with the treatment of HNF1-β antisense ODN (**Figures 7a-G and H**). The mRNA expression of collectrin and the genes under the control of HNF-1α and HNF-1β was investigated. Collectrin antisense ODN suppressed collectrin gene expression along with that of HNF-1, regulator of *Pkd2* and *Umod*. Notably, the expression of collectrin was inhibited by HNF-1β antisense ODN, however, inhibitory effect was not seen in HNF-1α antisense ODN treated group (**Figure 7b**). The addition of HNF-1β antisense ODN resulted in global inhibitory effects on HNF-1 regulated genes compared with HNF-1α antisense ODN treated metanephroi except *Tg737/Polaris.*

**Figure 7:** Collectrin antisense experiments in mouse metanephric organ culture system. *Panels aA & aB:* Addition of EGF (12.5 µg/ml) (EGF) into culture media induces hypertrophy of the fetal kidney without cyst formation compared with nonsense ODN (oligodeoxynucleotide)-treated control explants (CON). *Panels aC & aD:* The formation of cleft-like cysts (arrows) in the ureteric bud branches are seen in collectrin antisense ODN treated groups at concentrations of 1.5 µM (COLL-1.5) and 2.5 µM (COLL-2.5). *Panels aG & aH:* The formation of multiple cleft-like cysts is accentuated in metanephroi treated with HNF-β antisense ODN at concentrations of 1.5 µM (HNF-β-1.5) and 2.5 µM (HNF-β-2.5). *Panels aE & aF:* Similar effect, although somewhat less, is seen in HNF-1α antisense ODN treated group at concentrations of 1.5 µM (HNF-α-1.5) and 2.5 µM (HNF-α-2.5). *Panel b:* mRNA expression of collectrin and the genes regulated by HNF-1α and HNF-1β including *Pkhd1*, *Pkd2*, *Umod*, and *Tg737/Polaris*. Scale bars, 200 µm for panel a.

### Collectrin expression decreased in polycystic kidneys

To investigate collectrin expression and localization in cystic kidneys, we performed immunochemistry on the kidneys from HNF1βΔC transgenic mice. Transgenic mice at postnatal day-52 (P52) and P100 were compared with a non-transgenic littermate at P52. The kidney-specific expression of HNF1βΔC was associated with renal cyst formation and extensive interstitial fibrosis throughout the parenchyma of the kidney (**Figure 8a**). Collectrin was expressed in cytoplasm and apical membrane throughout collecting duct cells in the non-transgenic mice. In HNF1βΔC transgenic mice, weak apical expression was detected in morphologically normal collecting ducts, while the signals were barely detectable in single-layered or mutilayered cysts (**Figure 8b**). Collectrin in the kidney tissues from ADPKD patients was seen localized in morphologically normal tubules, whereas the epithelial cells lining single cell- and multi-layered cysts showed weak or lacked collectrin expression (**Figure 8c**).

**Figure 8:** Collectrin expressions in polycystic kidneys. *Panel a:* Kidney tissues from nontransgenic littermates at postnatal day 52 (P52), HNF1βΔC transgenic mice at P52, and HNF1βΔC transgenic mice at P100. Numerous renal cysts are formed in kidneys of HNF1βΔC transgenic mice. (Masson-Trichrome) *Panel b:* Immunoperoxidase staining of collectrin. Abundant expression of collectrin is seen in nontransgenic mice P52. Collectrin immunoreactivity is readily seen in normal portion of collecting duct cells (arrow head) but not seen in the epithelia lining the cysts (arrow) in HNF1βΔC transgenic mice. *Panel c:* Collectrin immunoperoxidase staining in kidney tissues form normal human and ADPKD patients. Abundant expression of collectrin is seen in normal collecting duct cells. In ADPKD patients, collectrin expression is observed in normal collecting duct cells (arrow head); however immunoreactivity of collectrin is not seen in both single-layered (arrow) and multilayered cysts. Scale bars, 1 mm for panel a, 50 µm for panels b and c.

## Discussion

In the kidney, HNF-1β, a transcriptional factor, has been shown to modulate activities of several target genes in tubular epithelia, namely *Umod*, *Pkhd1*, *Pkd2* and *Tg737/Polaris*. Mutations in these genes have been described in various forms of cystic diseases. Although HNF-1α and HNF-1β bind to the target site with similar affinities, either as homo- or hetero-dimers, the findings of the present study suggest that collectrin is another novel target of HNF-1β in the kidney. In the kidney tissues, HNF-1α was expressed exclusively in the nuclei of renal proximal tubular cells, while HNF-1β was expressed in all segments of the nephron, including collecting ducts[7]. Interestingly, the RT-PCR analyses revealed that both HNF-1β and collectrin are co-expressed in collecting duct and respective cell lines, including mIMCD-3, mIMCD-K2, RCCD1, RCCD2, and M-1 cells, suggesting a potential functional association between these two molecules. Besides kidney, collectrin is also co-expressed with HNF-1β in pancreatic islets[13], suggesting that the transcriptional activities are perhaps under tight and specific control of HNF-1β.

Many of HNF-1β driven proteins linked to PKD in mouse and human localize to the primary cilium[20], [21]. Cilia are rod-like organelles originating from the basal body and related to the centriole. Their basic structure consists of a central axoneme composed of 9 doublets of microtubules and a ciliary membrane that is continuous with plasmalemma. One to two primary cilia are present on the surface of most vertebrate cells and also on the apical surface of tubular epithelia of mammalian kidney[22]. A series of discovery began from an insertional mutagenesis screen in mice and the mutation in Tg737 gene was found to cause recessive form of PKD in *orpk* mice[23]. The protein product of *Tg737*, polaris, is localized in the axoneme and basal body. It seems to be essential for ciliary assembly and intra-flagellar transport[24], [25]. In addition to structural abnormalities of cilia, functional defects were noted in *Invs* [26] and *Cys1* [27], and both mouse mutants revealed ARPKD phenotype. Later studies revealed that the PKD1 product, polycyctin-1, as well as polycystin-2, polaris, and cystin are all found to be localized to primary cilia in cultured mouse cortical collecting duct cells[28]. Interestingly, defects in primary cilia are seen in Bardet-Biedl syndrome (BBS), characterized by mental retardation, pigmentary retinopathy, polydactyly, obesity, renal cyst formation and hypogenitalism. Among 8 causal genes, BBS8 protein localizes to centrosomes and basal bodies and co-localizes with γ-tubulin and BBS4[29], [30]. Although ciliary functions in renal tubules are incompletely understood, this organelle most likely functions as a flow-sensitive mechanosensor to luminal fluid flow, modulates flow-sensitive ion transport and possibly regulates cell proliferation and differentiation[31].

Like other genes involved in cystogenesis, it is reasonable to speculate that the HNF-1β-driven collectrin plays a role in ciliary functions and thereby in cystogenesis in PKD, since collectrin co-localized with acetylated α-tubulin, maker for primary cilium. In peri-basal body region of primary cilium, collectrin was seen surrounding basal body marker, γ-tubulin, and it revealed immunoreactivities on the microvesicle revealed by immunoelectron microscopy (**Figures 2** **and** **9**). Cilia and flagella are unable to synthesize the various ciliary proteins, and thus all non-membrane-bound proteins needed for elongation of the primary cilium are transported to the ciliary tip to endow it with functional properties[32], [33]. The process is accomplished by a transport apparatus known as the intraciliary or intraflagellar transport (ICT or IFT) system. In *Chalamydomonas*, the IFT particles are composed of at least 17 subunits; the IFT polypeptides move in antrograde direction to the flagellar tip by kinesin-II and move in the retrograde direction to the base of the flagellum by cytoplasmic dynein 1b[34]. However, it is not clear how integral membrane proteins are transported within cilia and flagella. Since some membrane proteins are concentrated in the ciliary membranes, the barrier has to exist at the base of cilium to prevent backward diffusion out of the cilium or one-way barrier facilitates the transportation of integral proteins from the apical plasma membranes[35] (**Fig. 8**); the former is rather conceivable and the base of the cilium would be expected to serve as an initial docking station[36].

**Figure 9:** Models for the trafficking of cilliary integral membrane proteins.

Snapin is a 15 kDa protein containing predicted coiled-coil domain in its C-terminal half[37] and it has been reported to bind to synaptic SNARE (soluble N-ethylmaleimide-sensitive-factor attachment protein receptor) complex via a direct interaction with SNAP-25 and SNAP-23 and thus is believed to be involved in vesicle fusion and trafficking[38]. Our previous studies suggest a direct binding between collectrin and snapin by yeast two hybrid system and GST-pull-down assay[13]. Furthermore, immunoprecipitation studies in pancreatic β cell line, INS-1 cell, indicated that collectrin binds to SNARE complex, consisting vesicle-associated membrane protein-2 (VAMP-2), syntaxin-1 and SNAP-25, via direct interaction with snapin[13]. Incidentally, the presence of SNARE proteins such as SNAP-23, syntaxin-4 and VAMP-2 has been reported in collecting duct cells[39]. The current studies extended the observations and demonstrated that collectrin co-immunoprecipitated with snapin and SNARE proteins, SNAP23 and syntaxin-4 in collecting duct cells. In addition, complex formation of collectrin with γ-actin, myosin II-A (non-muscle heavy chain II-A), and tropomyosin was elucidated. The interaction of actin with non-muscle myosin II-A assembled around aggregates of secretory vesicles facilitate their exocytosis in lacrimal acinar epithelial cells[40]. In other cell types, myosin II is involved in vesicle budding from Golgi[41], intracellular vesicle movement or trafficking[42]–[45], and membrane docking[40], [46]. In view of these processes described in other cell types and elucidated in this investigation, it would suggest that collectrin in association with SNARE and actin-myosin complex mediates specific vesicle transport and docking to drive the integral membrane proteins to ciliary membranes. In support of such a contention, the application of collectrin siRNA to mIMCD3 cells resulted in severe defects in cilium formation and subsequent loss of polycystin-2 on cilia, increased cell proliferation and apoptosis, and overexpression of EGFR and its mislocalization. This phenomenon is consistent with the facts that the presence of a cilium is associated with the establishment of polarity and differentiation of the cells in the stationary or G0 phase of the cell cycle. In many cells, the entry into the cell cycle is preceded by ciliary resorption; while exit from mitosis is accompanied by cilium formation[47].

Another significant finding of our study is that collectrin forms complex with polycystin-2 and *Tg737/Polaris*. Polycystin-1 is a G protein-coupled transmembrane receptor that acts as a ciliary mechanosensor and regulates calcium channel activities of polycystin-2. Polycystin-1 and -2 forms a hetrerodimer complex in primary cilium and polycyctin-2 responds to signals from polycystin-1 induced by the ciliary flexing to generate influx of calcium[31]. Polycystin-1 and polycystin-2 was co-localized both in apical and basolateral membranes including primary cilium, cell-cell adherens junction, and cell-matrix focal adhesion. In contrast to polycystin-1, the presence of polycystin-2 in endoplasmic reticulum (ER) and Golgi apparatus suggests that ER and Golgi are recycling pool or the site of polycystin-2 activity[48]. The trafficking of proteins to specific subcellular compartments is governed by multiple protein-protein interaction following post-translational modifications[49]. Polycystion-2 is phosphorylated on Ser812 by protein kinase (CK2), binds to phosphofurin acidic cluster sorting protein/Golgi-derived coat protomer I (PACS2/COPI), and is retrieved on the ER. Dephosphorylation of polycystin-2 by protein phosphatase 2A (PP2A) facilitates polycystin-2 translocation to the plasma membrane by releasing from the interaction with PACS proteins[50]. Similarly, the retrieval to the Golgi is mediated by PACS-1/adaptin. Other molecules that may modulate these events include CD2-associated protein (CD2AP) which participates in endocytosis of polycystin-2, while PIGEA-14 is involved in forward trafficking from the ER to the Golgi[51]. The above literature information can be interfaced with the current findings suggesting collectrin in association with polycystin(s) modulate the ciliary pathobiology. The application of collectrin siRNA into mIMCD3 cells reduced polycystin-2 expression and resulted in selective loss of polycystin-2 from primary cilium, apical membrane and cytoplasm. The collectrin expression in the Golgi apparatus and ER suggests that it may also be involved in the ER-Golgi-plasma membrane trafficking of polycyctin-2. Defective trafficking of the latter may be case in mice with *Tg737^orpk^* mutation where polycystin-2 is seen accumulated in the stunted cilium, since *Tg737/Polaris* is not required for moving polycystin-2 into cilia but is needed to recycle it to the cell body[52]. The findings of the present investigation indicating an association of collectrin and *Tg737/Polaris* may also suggest a possible role of collectrin in such intraciliary recycling events of integral transmembrane proteins.

In summary, it seems that collectrin is necessary for the maintenance of primary cilium to supply the primary cilia-specific integral membrane proteins, including polycystin-2, and it is involved in multiple membrane trafficking processes; vesicle transport, docking to base of primary cilia, ER-Golgi trafficking, and intraciliary recycling. Credence to this notion comes from the studies where suppression of collectrin expression resulted in severe defects in cilium formation in mIMCD3 cells and slit like cyst formation in mouse metanephric organ culture system. Furthermore, the reduction of collectrin expression in cystic tubular epithelia in HNF1βΔC transgenic mice as well as in human ADPKD patients would be supportive of the role of collectrin in cystogenesis. Lack of phenotype of cyst formation in collectrin knockout mice suggested that ACE2 may compensate of collectrin action. The findings of this study that collectrin plays a central role in pathways common to cystogenesis of various hereditary cystic diseases should yield an impetus to develop new therapeutic intervention for the treatment of PKD with collectrin being a novel target.
